The article "The Expressions and Functions of lncRNA Related to m6A in Hepatocellular Carcinoma from a Bioinformatics Analysis" was published in 2022. Journal: Comput Math Methods Med.

# The Expressions and Functions of lncRNA Related to m6A in Hepatocellular Carcinoma from a Bioinformatics Analysis

**DOI:** 10.1155/2022/1395557

**Published:** 2022-10-12

**Authors:** Shengwei Du, Ying Guo, Jian Huang, Jiajia Xu, Guorong Chen

**Affiliations:** The First Affiliated Hospital, Wenzhou Medical University, Wenzhou, China

## Abstract

Hepatocellular carcinoma (HCC) is one of the most common cancer in these days. Besides, N6-methyladenosine (m6A) plays an important role in the occurrence and development of hepatocellular carcinoma. Meanwhile, it is known to us that long noncoding RNAs (lncRNA) have the capability to control the expression of genes which means some lncRNA can adjust the expression of some m6A.Thus, it is indispensable to dig the m6A-related lncRNA in hepatocellular carcinoma about its potential regulatory mechanism and immune analysis as well as its potential drugs. In this experiment, expression profile and clinical information of lncRNA are obtained by downloading the liver cancer data set from The Cancer Genome Atlas (TCGA) database. GO enrichment analysis is used to predict potential regulatory mechanism of lncRNA. Correlation analysis of clinical parameters are calculated via chisq.test. The Cox regression model is used in univariate and multivariate analysis, and the difference is statistically significant when *P* < 0.05. The results show that many kinds of lncRNA have influence on the prognosis of patients with HCC, and enrichment analysis discloses some pathways that can be used to evaluate mechanism underlying in HCC. The screening of targeted drugs can provide new clues for further experiments and clinical treatment.

## 1. Introduction

HCC is a malignant hepatocellular tumor [1], which is usually divided into two categories: primary HCC and secondary HCC [2]. Primary malignant tumor of the hepatocellular originates from the epithelial or interstitial tissue of the hepatocellular [2]. It has a high incidence in China and is extremely harmful [1]. Secondary or metastatic HCC refers to the invasion of hepatocellular by malignant tumors originating from multiple organs of the body [3], which is less common than primary hepatocellular carcinoma. Treatments usually include surgery, chemotherapy, and radiotherapy [2]. Due to the asymptomatic early stage of HCC, many patients have been diagnosed with HCC close to advanced stage [1]. Because of the poor prognosis of advanced hepatocellular carcinoma, even new promising treatments, including targeted therapy and biotherapy, are difficult to achieve satisfying results [2]. The 5-year survival rate of Chinese patients diagnosed after stage Ib is less than 50% [4]. Therefore, it is necessary to find new treatment strategies and drugs. lncRNA is a nonprotein RNA fragment with a length of more than 200 bp [5]. According to its loci in the genome, it can be divided into antisense lncRNA, intron noncoding RNA, intergenic lncRNA, sense lncRNA, and bidirectional lncRNA [6]. It plays an important role in many biological processes such as chromatin interaction, transcriptional regulation [7], mRNA posttranscriptional regulation, and epigenetic regulation. lncRNA is also considered to be an emerging participant in promoting the initiation and progression of cancer in recent years [6] and plays an important role as a carcinogenic or tumor suppressor gene in the occurrence and development of tumors [8]. Studies have shown that abnormal expression, deletion, or mutation of lncRNA is closely related to the occurrence, development, and metastasis of hepatocellular carcinoma [9]. mRNA modification directly leads to protein changes and affects cell function, and studies have shown that mRNA methylation is a reversible and dynamic modification process [10]. Among them, N^6^-methyladenosine (m6A) modification is the most abundant form of methylation modification of mRNA [11]. m6A is widely involved in regulating all stages of the life cycle [12–16], including mRNA splicing, processing, translation, and degradation, and plays an important role in the progression of malignant tumors [17] . TCGA project is a large-scale sequencing genome analysis technology to map the genome of human tumors [18–20], including 33 types of cancers [21]. This study is based on HCC transcriptome data, clinical information, and mutant messages in the TCGA public database.

The article "The Expressions and Functions of lncRNA Related to m6A in Hepatocellular Carcinoma from a Bioinformatics Analysis" was published in 2022. Journal: Comput Math Methods Med.

## 2. Materials and Methods

### 2.1. Data Collection and Processing

Bioconductor/TCGA [22] biolinks function package to download the standardized and processed mRNA expression data, clinical messages, and mutant information of hepatocellular carcinoma data set from the TCGA database (https://tcga databases http://data.nci.nih.gov/tcga/) [23–26]. The total number from TCGA of samples of the original study is 424, containing 374 HCC samples and 50 nonplastic tissue samples.

### 2.2. Coexpression Analysis

Isolation of lncRNA from hepatocellular carcinoma transcriptome data by perl then utilizes “limma” package in *R* and extracts the expression of m6A followed by analysis of coexpressed between lncRNA and m6A as well as using “limma” package in *R*. And the expressions of m6A-related lncRNA are disclosed.

### 2.3. Construction of Prognostic Model

After merging the expression data of lncRNA which correlated with mRNA and survival statistics, the patients are randomly divided into train group and test group by “survival” packages and “survmiminer” packages of *R*, while calculating the median risk. Therefore, the patient can be divided into high-risk group and low-risk group according to median risk obtained above. In the basement of clinical information and risk score, survival curve and risk curve can be acquired. The risk coefficients of age, sex, tumor grade, tumor stage, and the risk score of the prognostic risk model are calculated by univariate regression analysis and multivariate regression analysis. The accuracy of the prognostic model erected above is judged by the area under the ROC curve (AUC), judging the relationship between clinical data, prognostic risk model, and survival time via *C*-index curve.

The article "The Expressions and Functions of lncRNA Related to m6A in Hepatocellular Carcinoma from a Bioinformatics Analysis" was published in 2022. Journal: Comput Math Methods Med.

### 2.4. GO(Gene Ontology) Enrichment Analysis and Immune Function Analysis

Referring the information of the GO database through the clusterProfiler package of *R* and org.hs.eg/.dbpackage of *R*, drawing GO enrichment plot by “enrichplot” package, “ggplot” package, “ggpubr” package, and “dplyr” package in *R*, and using “GSEABase” package from *R* to extract relevant data in the (Gene Set Enrichment Analysis) GSEA database and mapping a heat map of the changes connecting with immune function in hepatocellular carcinoma cells (HCC), the waterfall map of tumor mutation burden (TMB) in patients with hepatocellular carcinoma is painted relying on *R* package—“maftools.”

### 2.5. Data Analysis

Statistical analysis and graphic drawing are received by using *R*×64 4.1.0 software (https://www.r-project.org/) and univariate and multivariate analysis using the Cox regression model. The log-rank test is used to compare the survival rate in the high-risk group and low one. When the survival rate is estimated by Kaplan-Meier analysis, coxph function is used for Cox proportional hazard regression analysis, and chisq.test is used to analyze the relationship between clinical variables and prognosis of hepatocellular carcinoma patients. The difference is statistically significant when *P* < 0.05.

## 3. Results

### 3.1. Screening lncRNA Correlated with Prognosis and Coexpression with m6A

23 m6A and lncRNA which coexpress with m6A are screened out from the TCGA database, and then the relationship of m6A and lncRNA are described by Sanji diagram (Figure 1(a)). Each color represents one m6A on the top of the figure, and the width of different colors means the correlation between m6A and lncRNA. The wider the color is, the closer the relationship between m6A and LncRNA. Sanji diagram shows that YTHDC1, RBMX, and HNRNPA2B1 have more coexpressed lncRNA than others. However, a few lncRNA were coexpressed with YTHDF3 and ZC3H13. Then, removing the normal samples contained in data, the lncRNA expression and m6A expression are extracted and analyzed in order to get the heat map (Figure 1(b))which indicates that there is close relationship between AC010789.1 and METTL3, AC103760.1 and YTHDF3, AL158166.1 and YTHDF2, and MKLN1 − AS and YTHDF2. However, AL391832. 2and m6A screened out have no significant relation.

The article "The Expressions and Functions of lncRNA Related to m6A in Hepatocellular Carcinoma from a Bioinformatics Analysis" was published in 2022. Journal: Comput Math Methods Med.

### 3.2. Construction of Prognostic Model of lncRNA

Patients with HCC are divided into train group and test group. The median risk value is calculated by the survival time, state of HCC patients, and the expressive levels of lncRNA. The train group and the test group are divided into high-risk group and low-risk group, respectively, according to median risk value. Then, univariate regression (Figure 2(a)) constructed based on the process above, and every position of red square represents the hazard ratio (HR) of different lncRNA. We can clearly identify from the diagram that the risk values of LINC01515, AL137127.1, and EIF2AK3-DT are significantly correlated with the prognosis of patients with HCC, whose hazard ratio is 10.403, 9.138, and 8.767, respectively. In the basement of the constructed model, survival curve and risk curve can be constructed (Figures 2(b)–2(e)). It is obvious that with the increase of risk score, the survival time of patients becomes shorter, and the number of deaths increases. Kaplan-Meier analysis (Figures 3(a) and 3(b)) shows the overall survival time of patients. As we can see from Kaplan-Meier analysis, red point means deceased patient while blue point means patients whose living is obvious that with the increasing of the risk score, patients have less survival time (*P* < 0.05). Also, heat map (Figures 3(c) and 3(d)) of the lncRNA selected above suggests that the expression of AL391832.2, AL158166.1, AC010789.1, and MKLN1-AS in high-risk patients is higher than that in low-risk patients, but the expression of AC103760.1 adverse means it expresses more in low risk patients. And the model needs to be judged. Thus, ROC curve (Figures 4(a) and 4(b)) is painted, and it believes that the area under the concentration curve (AUC) predicted the 1-year overall survival time, 3-year overall survival time, and 5-year overall survival time of HCC patients are 0.751, 0.722, and 0.700, respectively. And AUC values of risk are 0.751 which is more than the AUC value of age, sex, tumor grade, and tumor stage. This implies that the risk model we constructed is more sensitive than other index.

### 3.3. Independent Prognostic Value of lncRNA Prognostic Risk Model

Univariate Cox regression analysis (Figure 5(a)) explains the hazard ratio of different indices, and the hazard ratio correlates with the prognosis. As is shown in the diagram, age, gender, grade of HCC, stage of HCC, and risk score of the model are concluded. Also, it shows that the tumor stage of patients (HR = 1.680, *P* < 0.001) and risk model (HR = 1.236, *P* < 0.001) are liable to be prognostic factor. Multivariate Cox regression analysis (Figure 5(b)) indicates that the tumor stage of patients (HR = 1.531, *P* < 0.001) and risk model (HR = 1.185, *P* < 0.001) are capable to be independent prognostic elements for hepatocellular carcinoma patients. Concordance index (*C*-index curve) (Figure 5(c)) depicts the relationship between index and prognosis of HCC patients over time. It is obvious that risk score whose *C*-index is beyond 0.7 is higher than age, gender, cancer stage, and grade, meaning that risk score is more closely related to prognosis of HCC patients. The clinical grouping model (Figures 5(d) and 5(e)) verifies that the survival rate of patients in stages I-II is different in the high-risk group and low -risk group meaning that patients in the low-risk group have more life span than those in the high-risk group. Interestingly, there is no significant difference between high-risk group and low-risk group in stage III-IV patients.

The article "The Expressions and Functions of lncRNA Related to m6A in Hepatocellular Carcinoma from a Bioinformatics Analysis" was published in 2022. Journal: Comput Math Methods Med.

### 3.4. Enrichment Analysis and Mutation Analysis

Gene Ontology (GO) (Figure 6(a)) analysis include biological process (BP), cellular component (CC), and molecular function (MF). As is shown in the picture, lncRNA is significantly enrich in collagen-containing extracellular matrix in CC, and lncRNA is collected in external encapsulating structure organization most in BP; as for MF, oxidoreductase activity, acting on paired donors, with incorporation or reduction of molecular oxygen, recruits many lncRNA. The analysis of immune function (Figure 6(b)) suggests there is an obvious difference in the function of type-II-IFN-response, MHC-class-I, and APC-costimulation between the high-risk group and the low-risk group. The waterfall diagram (Figure 6(c)) was obtained by mutant analysis, and it shows that TP53 mutation accounted for the highest proportion in the high risk group, and in TP53 mutation missense mutations accounted for a higher proportion, followed by frameshift mutations. As for the low-risk group (Figure 6(d)), CTNNB1 mutation accounted for the highest proportion (29%), of which the most common is missense mutation. The difference tumor mutation burden (TMB) analysis (Figure 7(a)) showed that there is no significant difference in mutation between the high-risk group and low-risk group. However, the survival probability (Figure 7(b)) differs in HCC patients with high-TMB and low-TMB, while the survival curve (Figure 7(c)) suggests that the high-risk group with high tumor mutation load has a lower survival rate.

The article "The Expressions and Functions of lncRNA Related to m6A in Hepatocellular Carcinoma from a Bioinformatics Analysis" was published in 2022. Journal: Comput Math Methods Med.

### 3.5. Immune Escape and Immunotherapy

Tumor Immune Dysfunction and Exclusion (TIDE) (Figure 8(a)) hints that there is no significant difference in tumor immune escape, effect of immune checkpoint blockade therapy, and regulatory factor of immune checkpoint blockade therapy of HCC between the high-risk group and low-risk group. Meanwhile, the potential drugs (Figures 8(b)–8(l)) of HCC are screened, and 11 drugs were obatined: A.443654, A.770041, AG.014699, AICAR AKT inhibitor VIII, AMG.706, ATRA, AUY922, axitinib, AZ628, and AZD.0530.

## 4. Discussion

High postoperative recurrence rate and chemotherapeutic drug resistance in patients with HCC are the main factors of high mortality in patients [1]. Therefore, reliable molecular markers and potential drugs for predicting the prognosis of HCC are of great significance in guiding the prognosis of patients [27]. Besides, enrichment analysis provides efficient clues for further exploration about the mechanism underlying in HCC. Dysregulation of m6A modification has been associated with many human diseases including cancer [28], and accumulative evidence has supported the correlation between aberrant cellular m6A and human cancer [16], such as endometrial cancer [29] and renal cell carcinoma [30], but the importance of m6A in cancers still remains unclear. It has been confirmed that multiple types of lncRNA are ubiquitous in cancer [6], such as breast cancer [31], prostate cancer [32], and HCC [33]. Also, lncRNA has diverse regulatory functions [34] which is being systemically characterized before [8]. In this study, by calculating information from the TCGA database, it is found that there is a coexpression relationship between m6A and lncRNA in HCC. This is consistent with the research of He et al. [8]. We prove that the lncRNA was related to the prognosis of patients with hepatocellular carcinoma via constructing the Cox proportional hazard regression model. Concerning to the results, maternally expressed gene 3 (MEG3) [35], imprinted lncRNA gene, has been proved to be a tumor suppressor gene in HCC [36]. Also, HULC [37] upregulated dramatically in HCC [38]. Former studies have shown that the five-year survival rate of HCC is low in most developed and developing countries [39] but by scoring the risk of patients with high risk and low risk of HCC, obviously, the higher the risk is, the shorter the survival time of the patients is. Univariate Cox regression analysis and multivariate Cox regression analysis on the independent prognostic value of risk mode were as follows. lncRNA prompts that the established lncRNA model can be used as a prognostic factor and independent prognostic factor for patients with HCC. Enrichment analysis revealed the potential mechanism of lncRNA involved in the progression of liver cancer. Mutation analysis infers the potential mechanism of high-risk and low-risk patients in HCC. Emerging studies have proved that gene mutation plays a very important role in the occurrence and development of tumors. Immunoassay deduces potential drugs for hepatocellular carcinoma, but the deficiency is that immune analysis can only analyze the effect of single drug, instead of the combination of tumor drugs. In a summary, this study explored the lncRNA associated with m6A in HCC and successfully predicted some potential pathways and drugs, which provided some directions and evidence for further study involved in the mechanism and treatment of HCC.

The article "The Expressions and Functions of lncRNA Related to m6A in Hepatocellular Carcinoma from a Bioinformatics Analysis" was published in 2022. Journal: Comput Math Methods Med.

## Figures and Tables

**Figure 1:** Screen prognosis-related lncRNA and prediction of coexpression between m6A and lncRNA, The coexpression of various lncRNA and m6A was revealed by Sankey diagram (a). The heat map (b) indicates the correlative tendency among m6A and lncRNA (^∗∗∗^*P* < 0.001; ^∗∗^*P* < 0.01; ^∗^*P* < 0.05).

**Figure 2:** Univariate regression analysis (a) suggests the association between lncRNA and the prognosis of HCC patients. Survival curves for the test group (b) and train group (c) of the constructed model before assuming the survival probability in the high-risk group and low-risk group.

**Figure 3:** Dot plot prompts the survival time and survival state along with the increasing risk of HCC patients in the test group (a) and train group (b). The heat map of the test group (c) and train group (d) points out the variable expression of different lncRNA in groups with high risk and low risk.

**Figure 4:** ROC curve represents the reliability of the risk model constructed above. The sensitivity of survival time of HCC patients are predicted by risk score (a), as well as the sensitivity of risk, age, gender, grade, and stage (b).

**Figure 5:** Independent prognostic value of the risk model of lncRNA. Forest map of univariate Cox regression (a) indicates that stage of HCC and risk score is the relevant prognostic factors, and the multivariate Cox regression (b) hint stage of patients and risk score is the independent prognostic issues of HCC. *C*-index (c) curve suggests that the risk score is the most sensitive factors among them, while survival curve of different stages indicates the survival probability of HCC patients.

**Figure 6:** Enrichment analysis and mutation analysis. Gene Ontology analysis (a) points out the enrichment degree in BP, CC, and MF in HCC. Via immune function analysis, a heat map (b) collected shows the mutant immune functions in HCC. The alternative types in different genes of HCC patients in the low-risk group (c) and high-risk group (d) are obviously various.

The article "The Expressions and Functions of lncRNA Related to m6A in Hepatocellular Carcinoma from a Bioinformatics Analysis" was published in 2022. Journal: Comput Math Methods Med.

**Figure 7:** Violin drawing (a) indicates the similarity between high-risk group and low one in TMB. Interestingly, patients with high TMB could not be compared to patients with low TMB in survival probability (b), and the high-risk group with high tumor mutation load has lower survival rate.

**Figure 8:** Violin drawing (a) hints there is no significance between high-risk group and low one in tumor immune escape, immune checkpoint depression, and the regulatory factor. Then, 11 promising drugs (b-l) are selected relying on potential targets.
